# A Torn ACL Mapping in Knee MRI Images Using Deep Convolution Neural Network with Inception-v3

**DOI:** 10.1155/2022/7872500

**Published:** 2022-02-08

**Authors:** S. Sridhar, J. Amutharaj, Prajoona Valsalan, B. Arthi, S. Ramkumar, S. Mathupriya, T. Rajendran, Yosef Asrat Waji

**Affiliations:** ^1^Department of Computer Science and Engineering, Saveetha School of Engineering, Saveetha Institute of Medical and Technical Sciences, Chennai, India; ^2^Department of ISE, RajaRajeswari College of Engineering,Mysore Road, Bangalore, Karnataka, India; ^3^Dhofar University, Salalah, Oman; ^4^Department of Computer Science and Engineering, College of Engineering and Technology, SRM Institute of Science and Technology (Deemed to Be University), Kattankulathur, Chennai, Tamilnadu, India; ^5^Department of Computer Applications, Kalasalingam Academy of Research and Education (Deemed to Be University), Srivilliputhur, Tamilnadu, India; ^6^Department of Computer Science and Engineering, Sri Sairam Institute of Technology (Autonomous), Chennai, Tamilnadu, India; ^7^Makeit Technologies (Center for Industrial Research), Coimbatore, Tamilnadu, India; ^8^Department of Chemical Engineering, College of Biological and Chemical Engineering, Addis Ababa Science and Technology University, Addis Ababa, Ethiopia

## Abstract

The anterior cruciate ligaments (ACL) are the fundamental structures in preserving the common biomechanics of the knees and most frequently damaged knee ligaments. An ACL injury is a tear or sprain of the ACL, one of the fundamental ligaments in the knee. ACL damage most generally happens during sports, for example, soccer, ball, football, and downhill skiing, which include sudden stops or changes in direction, jumping, and landings. Magnetic resonance imaging (MRI) has a major role in the field of diagnosis these days. Specifically, it is effective for diagnosing the cruciate ligaments and any related meniscal tears. The primary objective of this research is to detect the ACL tear from MRI knee images, which can be useful to determine the knee abnormality. In this research, a Deep Convolution Neural Network (DCNN) based Inception-v3 deep transfer learning (DTL) model was proposed for classifying the ACL tear MRI images. Preprocessing, feature extraction, and classification are the main processes performed in this research. The dataset utilized in this work was collected from the MRNet database. A total of 1,370 knee MRI images are used for evaluation. 70% of data (959 images) are used for training and testing, and 30% of data (411 images) are used in this model for performance analysis. The proposed DCNN with the Inception-v3 DTL model is evaluated and compared with existing deep learning models like VGG16, VGG19, Xception, and Inception ResNet-v28. The performance metrics like accuracy, precision, recall, specificity, and F-measure are evaluated to estimate the performance analysis of the model. The model has obtained 99.04% training accuracy and 95.42% testing accuracy in performance analysis.

## 1. Introduction

ACL tear is a typical physical problem among young athletes with an annual occurrence of 0.8 per 1000 in the general population but as high as 100 for professional football players for every 1000. With the noncontact loading of a valgus knee, ACL injuries most commonly occur when turning the other direction, causing a constrained internal rotation of the tibia [1].

ACL tear might be partial and completely teared. Partial tear ranges from the small tears, including only few fibres, to a high-grade, near, and complete tear including practically the entire ACL fibres. A partial tear can include both or just a single bundle to a varying degree. In some cases, the plastic deformity of the ACL without fiber discontinuity can cause ACL insufficiency [2]. ACL tear detection depends on assessing the obliquely oriented structures on several images segments with various tissues contrast utilizing the integration of MRI discoveries such as discontinuity of fiber, contour changes, and abnormality of signal inside the injured ligaments [3].

Over the past decade, the role of imaging in osteoarthritis (OA) research has grown significantly. Magnetic resonance imaging (MRI) was one of the key components of large-scale longitudinal tests, providing a rich array of musculoskeletal tissue functional and structural characteristics that were previously unavailable. It is necessary to improve data management, quality assurance, automated postprocessing images pipelines, and multidimensionality feature space dissection methods in order to make better use of this data resource, which comes at a higher cost and contains more perplexing quantitative information volume [4]. When examining the tear in the ACL, the coronal, sagittal, and axial planes are taken into consideration. When the ligaments were first detected on the sagittal planes, they were followed from distal to proximal in order to evaluate where the rip had occurred. As a result, the sagittal and coronal planes were thoroughly analyzed in order to confirm the presence of the teared region. As soon as the spirally teared pattern was recognized, the middle part of the spiral was designated as the teared region [5].

MRI is a sort of medical imaging that is believed to be a successful method due to the fact that it is noninvasive and that it has superior soft-tissue contrast compared to other types of imaging. When compared to ionizing radiation-based methods, it does not alter the structure, construction, or properties of particles in the way that they do. As a result, magnetic resonance imaging (MRI) can provide a wealth of information on tissue structures, such as their size, shape, and location. Massive amounts of attention are drawn to magnetic resonance imaging (MRI) for medical procedures and CADe (computer-aided detection) [6].

Furthermore, the two factors that had the biggest impact on the results of medical image processing and analysis were the picture acquisitions and the image interpretations. It is commonly known that improved image quality leads to better results when photographs are processed, and this is true in this case. In many circumstances, the image quality was dependent on the quality of the image acquisition; in this way, better image acquisitions resulted in higher image quality overall. Not only does magnetic resonance imaging (MRI) have the advantages of being noninvasive and providing superior soft-tissue contrast, but it also does not expose patients to high levels of ionizing radiation. As a result, magnetic resonance imaging (MRI) could provide useful information about tissue structures; it is essential in medical image processing. As a result, MRI scans are the primary focus of this investigation. It is necessary to develop an image interpretation system that integrates a variety of functions such as image detection, segmentation, registration, and classification in order to obtain exact picture interpretation results. The deep learning model was used in this study in order to obtain the desired system.  Figure 1 shows the difference betwwenNormal and torn ACL in MRI.

Deep learning (DL) is the subcategory of machine learning approaches in artificial intelligences (AI). If the number of layers increases in the network, it is known as deep learning. It is additionally called deep neural network (DNN). It can learn from unstructured data, likewise by utilizing fine-tuning that is done by the backpropagation approach. Deep learning might be utilized to discover features automatically from the provided dataset for each particular application [7, 8]. Inspired by the effective and reliable execution of deep learning systems, DCNN was implemented for MRI medical images classification to classify ACL ligament tears.

In this research, an Inception-v3 DTL model based on DCNN was proposed for the classification of ACL tear using MRI images. The most important aspect of this study was the detection of an ACL tear from MRI knee image, which could be beneficial in determining the nature of a knee anomaly. Data preparation is the first stage of the process. During preprocessing, noise and other artifacts were eliminated from the images, and the images were adjusted to be suitable for the intended classification work. Following the preprocessing stage, the next step is to extract the features of the image. To carry out this research, the Inception-v3 DTL model was employed, which extracted features from an input preprocessed image and then delivered those features to a DTL model for training. The model that was created as a result of this training was eventually put to the test by deploying the DCNN classification model to distinguish between images of normal and abnormal (torn) ACL. Finally, the proposed model's performance was compared to those of other existing models for validation.

ACL tears and their associated complications are covered in this section, which serves as an introduction to the topic. In the next sections, related works will be covered in Section 2, the proposed methodology will be discussed in Section 3, the experimental analysis of results will be discussed in Section 4, and the conclusion and future directions will be discussed in Section 5.

## 2. Related Works

Valentina Pedoia et al. used 3D CNN to detect and stage the severity of patellofemoral and meniscus joint cartilage morphological degenerative alterations in patients with osteoarthritis and anterior cruciate ligament rupture. The deep-learning pipeline in this model is comprised of segmenting cartilaginous and meniscus tissue and classifying lesions within the region of the tissue that has been segmented. The U-Net model was employed for automatic segmentation, and a “shallow” 3D CNN was used for the staging and identification of the severity of meniscus lesions. The conventions that were used for architectural visualization were very similar to those that were used for U-Net. The feature maps that were obtained were flattened into one-dimensional vectors and then used as inputs to a fully connected layer that created class probabilities based on the features that were obtained. A random forest was trained to make the final forecast after the probabilities were merged with demographic characteristics and coupled with the final prediction.

A DCNN classification approach based on three distinct CNN approaches for detecting ACL tears was proposed by Fang Liu et al., who used DenseNet, VGG16, and AlexNet to detect ACL tears. In this model, the classification models had to be trained separately, which resulted in a high training burden. In addition, the training y was inefficient, which can be improved with more practice. In general, the classification and detection of structural abnormalities present in the isolated ligament were performed correctly, and the results were satisfactory.

Rehan Ashraf et al. proposed a DCNN model for big data medical image classification using MRI images of various organs and tissues, which was tested in a real-world environment. The DCNN was used to carry out the feature extraction and classification steps in this particular model. An approach based on GoogleNet's pretrained GoogleNet layer classifier was used to extract the features, and a softmax layer classifier was used to extract deep features. A total of 144 layers, including convolution and fully connected layers, were used. When comparing the performance analyses from different classes, the model attained an overall accuracy of 98 percent in total.

Christoph Germann et al. employed the DCNN to diagnose ACL tears in MRI images as well. Using homogenous versus heterogeneous knee MRI cohorts with varied pulse sequenced methods and variable magnetic field strengths, a performance comparison was seen in this study [9], which compared the performances of the two groups.

Milica M.B. and Marko C.B. created a brain tumor classification algorithm based on CNN using MRI scans, which they believe will be successful. This model was proposed to classify three types of cancer in the brain tumor, and it was found to be effective. To obtain distinct viewpoints, the MRI scans were obtained in three separate planes: axial, coronal, and sagittal. Images with T1-W contrast enhancement were used to do the classification, which was done by comparing images from different databases. According to this model, CNN performed well with an accuracy of 97.28 percent when using 60 percent of training and 20 percent of validation and 20 percent of testing data. While taking additional approaches into consideration, it is possible to improve the generalization capability of the network [10].

CMAK Zeelan Basha employed machine learning methods to automate the classification of MRI images in this research. Using this model, a novel MRI image classification approach was developed for recognizing self-activation descriptions, which was then used to provide specialists and radiologists with a well-ordered selection devising result. In order to remove noisy data, a Gaussian filter was utilized, and the FCM technique was used for partitioning the data. The statistical features were retrieved with the use of mean, kurtosis, and median values, and the PNN, SVM, and K-NN algorithms were employed for classification. SVM with statistical characteristics outperformed the other two algorithms in terms of accuracy, with 93.1 percent accuracy [11].

In [12], a model for categorization and identification of anomalies in MRI brain images was suggested, which makes use of convolutional neural networks. A CNN containing feature maps that had been preprocessed in the curvelet domain was employed for MRI classification. Because of its multidirectional capability, the curvelet gave a good sparse representation, and the features recovered were more exact than those obtained using other standard methodologies. The accuracy of this curvelet domain combined with CNN was improved during the training and validation processes [12].

According to [13], a DCNN model has been developed for comparing the diagnostic interchangeability and image quality of nonaccelerated images to 15-layered DCNNs or 3-layered CNNs images with the optimal number of layers for a sixfold acceleration of the knee MRI dataset, with the optimal number of layers being three.

Mazhar Javed Awan et al. suggested an automatic detection algorithm for ACL tears based on deep learning techniques. In this study, two models of CNN technique were used, one of which was a regular CNN model and the other was a customized CNN model. ACL MRI pictures were classified using a conventional model with five layers and a customized model with eleven layers. Both models were tested for classification using ACL images. According to [14], the modified CNN model has produced superior results than the regular CNN model in terms of learning rate, accuracy, and other factors.

## 3. Proposed Methodology

A DCNN model with pretrained Inception-v3 is proposed in this research. This Inception-v3 model is based on DTL as it is proposed to identify the ACL ligament tears from the input dataset by classifying the MRI scan images. To extract features from the dataset, a pretrained Inception-v3 model is used, and the DCNN model is used for classification. 299 × 299 × 3 is the input image resolution. DCNN usually performs well with a larger dataset over a smaller one. TL could be useful in the CNN applications where the dataset is not huge [13]. For applications with comparatively smaller datasets, the concept of TL utilizes the learned model from large datasets such as ImageNet. This removes the need for a large dataset and decreases the lengthy training time as needed when generated from scratch by the deep learning algorithm. TL is a deep learning method that uses the model trained for the single assignment as ainitial point to train the model for a similar assignment. It is typically much quicker and simpler to fine-tune a network with TL than training a network from scratch. By leveraging standard models that have already been trained on large datasets, it allows training models using similar small labeled data. Training time and computing resources can be significantly decreased. With TL, the model does not need to be trained for as many epochs (a complete training period on the entire dataset) like a new model.

There are many kinds of transfer learning; an effective way was to initialize from pre-rained models the parameters of deep architectures and thus fine-tune learning parameter for making it adaptable for the target domains. This technique was used if the dataset was smaller, and, related to feature spaces or tasks, the target domains shared similarities with the domain sources. In image, lower-level characteristics were generally among various classes of image like edges, curves, gradients, and so on; thus higher-level features were classes-specific. The pretrained deep architecture for the classifications of ACL MRI images was modified based on this assumption. TL is an efficient way of achieving meaningful results in classification issues with small data size. Also, the hypertuning of DTL models will further enhance the performance. A DTL model-based Inception-v3 is implemented in this work. The proposed model is used for feature extraction by utilizing its learned weights on the ImageNet dataset together with a convolution neural network. The proposed DCNN technique with Inception-v3 architecture for the classification of ACL images is shown in Figure 2.

Inception-v3 based DCNN model is considered for retraining; this model consists of AvgPool, convolution, maxpool, concat Layer, dropout, fully connected layer, and softmax function.

### 3.1. Average Pooling

It is a 2-dimensional (2D) function with a pool size of (8 × 8), which decreases the data variance and the computational complexity. This layer allows the outcome to flow to the next layer.

### 3.2. Convolution

A 299 × 299 × 3 input size is used by convolution function, and this layer generates the feature maps through convolving the input data.

### 3.3. Maxpool

It is a two-dimensional maxpooling function and it reduces the variance at data and the computational complexity. The maxpooling is used to extract essential features such as edges, and average pooling is used to extract features smoothly.

### 3.4. Concatenation

This layer is used to concatenate its several input blobs into a single blob of output, and it takes a list of tensors as the input, where all have the same type of shape expect concatenation axis. It returns an output of a single tensor while concatenating all the inputs.

### 3.5. Dropout

It is considered as the regularization approach to minimize overfitting in the ANNs by overcoming complexed coadaptations from the training data. Here, the dropout scale is considered as 0.4, and it was the very effective method for executing averaging with the neural network model. Moreover, dropout refers to dropout of the units such as visible and hidden sides in a considered neural network.

### 3.6. Fully Connected

This is used to connect all neurons to one layer and another layer, which works based on a conventional multilayer-preceptor (MLP) neural network.

### 3.7. Softmax

The softmax function is used like the output function, which works similarly to maxlayer when it was variable for training via gradient descents. The exponential functions would cause an increment in the probability of preceding layers and compared to the other values; correspondingly, all output summations will always be equal to one [15].

In general, a two-dimensional plane can form many independent neurons, and the DCNN was made of several layers in which multiple 2D feature mapping planes structure. There are four core segments of the DCNN. The first segment was the local perceptions that the global image does not need to be interpreted by each neuron in neural networks, yet just local and global information waacquired by collecting local data. Next was the method of convolutions. The convolution functionality which was for extracting features of image is shown in Figure 3, and, by using convolution kernel, the total parameters could be reduced higher. Weight sharing is third. It means that parameters of the similar convolution kernels were utilized for the entire image and because of different positions in an image, the weights in the convolution kernels would not be modified. In addition, convolution operations' weight sharing will significantly reduce the parameters of the convolution kernel. Pooling is the final segment. The pooling layer was normally set in the CNN behind the convolution layer, which could be utilized for decreasing feature dimensions of the performance of previous layer's convolution layer, simultaneously to retain adequate key images information details.

To evaluate the dot products of the weights and the values in the input, a filter, which was an array of weights, was used in a convolutional layer, which slides over the input from a previous layer. These weights are discovered through the process of backpropagation of errors. After applying an activation function that incorporates element-wise nonlinearity, a feature map is produced, with each entry representing an individual neuron output from a tiny local region of the input. The feature map was then used to train a neural network.

As filters are considered, if the number of filters is higher, then it is possible to extract more feature mappings, and the better the model performances are. The comparative trails of 32-32-64, 32-32-32, 64-64-64, and 64-64-128 filters were therefore used for selecting the most appropriate filters on the conditions that both resources of computing and DCNNs network performances were considered on holding the different hierarchical structures and various influencing unchanged factors. 64-64-64 was therefore chosen as convolution layer filters, considering the performance considerations, and every receptive field size is 5 × 5 [16].

In the case of Inception-v3, the probability of every label *k* ∈ {1,…, *K*} for every training example is calculated by

(1) $$\begin{array}{c} Q\left(k\;|\;z\right)=\frac{\text{exp}\left(y_{k}\right)}{\sum_{i}^{K}\text{exp}\left(y_{i}\right)}, \end{array}$$

where *y* represents the nonnormalized log probabilities. Distribution of ground truth over labels *p(k | z)* was normalized; hence, that ∑_*k*_*p*(*k* *|* *z*)=1. For this system, the loss was provided by cross-entropy:

(2) $$\begin{array}{c} C=\sum_{k=1}^{K}\log\left(q\left(k\right)\right)p\left(k\right). \end{array}$$

For logits yk, the cross-entropy loss is differentiable and can therefore be used for deep model gradient training, where the gradients have the simple form of ∂*C*/∂*y*_*k*_=*q*(*k*) − *p*(*k*), bound between −1 and 1. Normally, this means that the log-probability of the correct label is maximized when the cross-entropy is minimized. Thus, it can produce few overfitting issues. Inception-v3 considered the distributions over label with a smooth parameter ∈ independent of training examples *v(k),* where, for training instance, the label distributions *p*(*k* *|* *z*)=∂_*k*,*z*_ were exchanged by

(3) $$\begin{array}{c} {p^{\prime }}^{\left(k\;|\;z\right)}=\left(1-\epsilon \right)\partial_{k,z}+\epsilon v\left(k\right), \end{array}$$

which is a mixture of the original *p*(*k* | *z*) distribution with 1- ∈ weights and the *v(k)* fixed distribution with ∈ weights. For a uniform distribution *v(k)* *=* *1/K*, the label-smoothing regularization was applied such that it becomes

(4) $$\begin{array}{c} p{{}^{\prime }}^{\left(k|z\right)}=\left(1-\varepsilon \right)\delta_{k,z}+\frac{\varepsilon }{K}. \end{array}$$

Alternately, this could be interpreted like cross-entropy as

(5) $$\begin{array}{c} H\left(p{}^{\prime },q\right)=-\sum_{k=1}^{K}\log\left(q\left(k\right)\right)p{{}^{\prime }}^{\left(k\right)}=\left(1-\epsilon \right)H\left(p{}^{\prime },q\right)+\epsilon H\left(v,q\right). \end{array}$$

On the activation layer, there are several activation features, such as sigmoid, ReLU, and softmax. Its functionality was to combine nonlinear factors for improving the model's conditions; hence it needs to be nonlinear. The activation function of the sigmoid function can be expressed as

(6) $$\begin{array}{c} f\left(x\right)=\frac{1}{1+e^{-x}}. \end{array}$$

The activation function of ReLU is expressed as follows:

(7) $$\begin{array}{c} f\left(x\right)=\left\{\begin{array}{cc} 0, & x\leq 0,\\ x, & x>0. \end{array}\right. \end{array}$$

The activation function of the softmax layer is expressed as follows:

(8) $$\begin{array}{c} f\left(x_{j}\right)=\frac{e^{x_{j}}}{{\sum e^{x_{i}}}^{}}. \end{array}$$

In these above equations, *f(x)* is the activation function, and *x* is the activation function input.

It is a nonlinear function like ReLU or sigmoid, which is applied to the elements of a convolution and was known as the activation function. When one or more pooling layers were deployed to the feature maps generated by the convolutional layers, the computational difficulty of a CNN was reduced. This was accomplished by decreasing the size of the maps created by the convolutional layers. The methods of maximum pooling and average pooling are the most widely utilized. The output layer has as many nodes as the number of classes in the dataset, which was one hundred. The output was classified using the softmax function, which was implemented in the proposed work. The number of epochs defines the number of times that the neural network will be trained and validated before it is performed. It may take thousands of epochs for an algorithm to converge on a set of weights that provides an acceptable level of accuracy. In neural network's training and validation, the batch size is defined as the number of samples in the dataset that will be loaded and propagated throughout the training and validation of the neural network.

The learning rate regulates the size of weight and bias changes in the training algorithm's learning as it progresses. It was the value that should be specified at the level low enough to allow the neural network to converge while also being high enough to avoid spending an excessive amount of time training it. Hidden layer count refers to the number of FC layers in the neuron which have a specified weight for every identified neuron, which was updated as the training durations are completed. Every neuron has an activation value, which was determined depending on the values of its inputs and the weights assigned to them. When this calculation was completed, it returns a value that was used as input for the final layer, which uses the softmax function to classify MRI images into two categories: normal and torn ACL.

## 4. Performance Analysis

The performance analysis of the proposed DCNN with the Inception-v3 model is assessed using the dataset in this section. The model was evaluated using parameters such as accuracy, precision, recall, specificity, and F-measure. Also, a comparative analysis was conducted for the validation of the model proposed. The output is compared to other current deep learning models used for classification, such as VGG16, VGG19, Xception, and Inception ResNet-v28. On the MATLAB 2019a Simulink toolbox, all the experiments are implemented and carried out. The dataset is split into 70 percent for training and 30 percent for testing the performance analysis.

### 4.1. Dataset Description

The dataset used in this work is collected from the MRNet database. It is an open-access database for the knee MRI dataset. It can be downloaded from https://stanfordmlgroup.github.io/competitions/mrnet/site.

The MRNet dataset includes 1,370 knee MRI images diagnosed at Stanford University Medical Center. There are 1,104 (80.6%) abnormal images, 319 (23.3%) ACL tears, and 508 (37.1%) meniscal tears in this dataset; labels were acquired from clinical reports through manual extraction.

Acute and chronic pain, follow-up or preoperative assessment, and injury/trauma are the most common indications for knee MRI examinations included in this dataset. GE scanners (GE Discovery, GE Healthcare, Waukesha, and WI) were used for examination with a regular knee MRI coil and a routine noncontrast knee MRI protocol that included the following sequences: coronal T1 weighted, sagittal proton density (PD) weighted, axial PD weighted with fat saturation, coronal T2 with fat saturation, and sagittal T2 with fat saturation. A total of 775 (56.6%) used a 3.0 T magnetic field; the remaining used a 1.5-T magnetic field for examination. This model uses 70% of data (959 images) for training and testing and 30% of data (411 images) for performance analysis [17, 18].

### 4.2. Performance Metrics

The proposed DCNN with the Inception-v3 DTL model is proposed in this research and compared with deep learning models like VGG16, VGG19, Xception, and Inception ResNet-v28. The performance metrics like accuracy, precision, recall, specificity, and F-measure are evaluated to estimate the performance analysis of the model. For every validation, both training and testing results are evaluated and compared. The primary objective of this research is to detect the ACL tear from MRI knee images, which can be useful to determine the abnormality of the patient. The result of this model can be based on the outcome detected as normal or abnormal. The true positive, true negative, false positive, and false negative are correctly analyzed to estimate this model's outcome [19–21].

  True Positive (TP): It represents the total correct predictions in abnormal cases.
  False Positive (FP): It represents the total incorrect predictions in abnormal cases.
  True Negative (TN): It represents the total correct predictions in normal cases.
  False Negative (FN): It represents the total incorrect predictions in normal cases.

Accuracy is the model's estimation of the performance subset. It is the primary output metric used to calculate the efficiency of the classification process. It is usually used to estimate when both the positive and negative classes are equally important. It is calculated using the following equation:

(9) $$\begin{array}{c} \text{Accuracy}=\frac{TP+TN}{TP+TN+FP+FN}. \end{array}$$

Precision is a positive predictive value. The preciseness of the classification model is calculated using it. It is the measure of the cumulative predictive positive value of the correctly predicted positive observation. The lower precision value reflects that a large number of false positives affected the classification model. The measure of precision can be computed using the following equation:

(10) $$\begin{array}{c} \text{Precision}=\frac{TP}{TP+FP}. \end{array}$$

The sensitivity is also referred to as recall. It is the proportion of correctly predicted positive observation of the overall positive predictive value. The lower recall value reflects that a large number of false-negative values affected the classification model. The recall estimation can be calculated using the following equation:

(11) $$\begin{array}{c} \text{Recall}=\frac{TP}{TP+FN}. \end{array}$$

As per this model, specificity is the prediction that healthy subjects do not have an abnormality. It is the percentage of subjects with no injury/trauma that is tested as abnormal. The specificity estimation can be calculated using the following equation:

(12) $$\begin{array}{c} \text{Specificity}=\frac{TN}{TN+FP}. \end{array}$$

The F-measure estimates the accuracy of the test and is defined as the weighted harmonic mean of the precision of the test and the recall. The accuracy does not take into account how the data is distributed. The F-measure is then used to manage the distribution problem with accuracy. The F-measure estimation can be calculated using the following equation:

(13) $$\begin{array}{c} F-\text{measure}=\frac{2\times \text{Precision}\times \text{Recall}}{\text{Precision}+\text{Recall}}. \end{array}$$

As shown in Tables 1 and 2, the proposed DCNN-Inception-v3 model achieved better performance in training and testing for classifying the ACL tear MRI images. The model obtained 99.04% training accuracy and 95.42% testing accuracy, which is 3.1% to 9.9% increased performance compared to the other existing compared models. VGG16, VGG19, Inception ResNet-v28, and Xception achieved 95.13%, 95.66%, 90.74%, and 92.48% in training and 85.45%, 87.90%, 89.91%, and 92.25% in testing performance, respectively. Inception-ResNet-v28 and Xception model achieved better performance in testing compared to the training performance. The performance was the same as accuracy for other parametric evaluations like recall, precision, specificity, and F-measure.

Compared with both testing and training results, the VGG16 approach achieved the least performance in every parameter, and the Xception model has achieved close results to the proposed model. The graphical chart of the comparison is plotted in Figures 4 and 5.

## 5. Conclusion

In this research, a DCNN based Inception-v3 DTL model was proposed for classifying the ACL tear MRI images. The proposed model was executed in four stages. Data preprocessing is the initial stage. After preprocessing, the next stage is to extract the features of image and then to deliver the features extracted into the model to train. The trained model was finally tested. The dataset used in this work was collected from the MRNet database. It is an open-access database for the knee MRI dataset. A total of 1,370 knee MRI images were used for evaluation. 70% of data (959 images) were used for training and testing and 30% of data (411 images) were used in this model for performance evaluation. The proposed DCNN with the Inception-v3 DTL model was assessed and correlated with existing deep learning models like VGG16, VGG19, Xception, and Inception ResNet-v28. The performance metrics like accuracy, precision, recall, specificity, and F-measure were evaluated to estimate the performance analysis of the model. For every validation, both training and testing results were evaluated and compared. The model has obtained 99.04% training accuracy and 95.42% testing accuracy, which was 3.1% to 9.9% higher than the other existing compared models in performance. However, this model was proposed to classify the ACL tear injuries from knee MRI images and has obtained better results in validation. In the future, the proposed model can be used to find any abnormalities present in various body organs by using different datasets like a brain tumor, heart disease, lung cancer, and so forth. The performance can be further increased by implementing a new deep transfer learning model with better classification performance.

## Figures and Tables

**Figure 1:** Difference between normal and torn ACL in MRI.

**Figure 2:** Proposed model.

**Figure 3:** Architecture of the proposed model.

**Figure 4:** Graphical plot of performance analysis of training.

**Figure 5:** Graphical plot of performance analysis of testing.

**Table 1:** Performance analysis of training evaluation.

Models	Accuracy	Precision	Recall	Specificity	F-measure
VGG16	95.13	95.05	94.64	96.25	94.72
VGG19	95.66	94.22	94.80	96.90	95.39
Inception ResNet-v28	90.74	89.90	89.26	91.72	90.56
Xception	92.48	91.94	91.67	93.36	92.07
Proposed	99.04	98.96	98.45	99.18	98.81

**Table 2:** Performance analysis of testing evaluation.

Models	Accuracy	Precision	Recall	Specificity	F-measure
VGG16	85.45	85.74	84.23	85.67	85.19
VGG19	87.90	87.50	86.06	88.72	86.09
Inception ResNet-v28	89.91	89.32	88.35	90.43	89.24
Xception	92.25	91.48	91.29	93.11	91.92
Proposed	95.42	95.02	95.13	96.34	94.83

## Data Availability

The datasets used and/or analyzed during the current study are available from the corresponding author upon reasonable request.
